The article "Study on Strength and Quality Training of Youth Basketball Players" was retracted in 2023. Reasons: signs of a paper mill; suspected computer-generated content; unreliable results or conclusions; lack of ethics approval or compliance.

# Study on Strength and Quality Training of Youth Basketball Players

**DOI:** 10.1155/2022/4676968

**Published:** 2022-08-18

**Authors:** Qinghui Meng

**Affiliations:** Shanxi University, Taiyuan City, Shanxi Province 030006, China

## Abstract

In order to scientifically explore the effective path of strength quality training of basketball players and improve the effect of strength quality training of basketball players, this paper takes young basketball players as the research object and comprehensively observes the changes and improvement of strength quality by building a strength training monitoring system for basketball players. On this basis, it is proposed to integrate blood flow restriction and basketball players' special strength training. Through the comparison with the traditional resistance strength training method, it is found that after 8 weeks of experimental comparison, the athletes' strength quality test indicators show that the average 3RM of the experimental group 1 bench press is 65.2 kg, the experimental group 2 is 65.7 kg, and the experimental group 3 is 72.2 kg. The average performance of the traditional control group was 55.4 kg. Compared with the traditional group, the average performance of the three experimental groups in bench press was significantly improved, which also verified the feasibility of this method in strength quality training.

## 1. Introduction

Any sports event is completed by the muscle tissue as an active sports organ with different compliance intensity and contraction speed and then drives the movement of bones of specific sports organs to complete the action. If the strength brought by the contraction and relaxation of human muscles is improved in the process of sports, the effect of sports is bound to be affected. The running, jumping, and confrontation in the process of sports are inseparable from the strength quality of athletes, and a good strength quality will have a higher sports effect. Especially for basketball players, because basketball itself is a competitive sport, basketball players will face a lot of physical confrontation in the process of competition [1, 2]. Physical confrontation must rely on good strength quality as support, so special strength training of athletes is very important. This paper introduces a blood flow restriction training method and discusses the feasibility of special strength training by comparing with traditional resistance strength training.

## 2. Literature Review

Leng et al. analyzed the impact of core strength training on swimmers through empirical research. The results show that athletes can effectively improve their core strength through a period of core strength training. When athletes make various technical actions, they can greatly improve the coordination between the muscle groups involved, which is conducive to athletes' better control of the body's focus, so as to improve athletes' special technical ability and improve their sports performance [3]. Gómez-Carmona et al. conducted empirical research on the core strength training of fencing athletes. The research shows that fencing athletes can significantly improve their core strength, core endurance, core explosive power, and other abilities after a period of training by choosing their own core strength training methods [4]. Zou et al. conducted core stability training experiments on track and field athletes. The results of the experiments show that after receiving a period of core stability training, middle- and long-distance runners can greatly improve their running efficiency and respiratory muscle ability and effectively reduce the probability of athletes' sports injury [5]. Li and Wang believe that because core strength training plays an important role in the performance of throwing athletes, athletes can significantly improve their body coordination and flexibility after a period of core strength training and maximize the strength of all parts of athletes [6]. Mwanzia et al. believe that in modern basketball, athletes need to have good core strength quality as support and guarantee when making basic technical actions such as moving, shooting, changing direction, passing, and breakthrough [7]. Only basketball players have strong core strength quality; they can ensure the stability of their bodies when making various technical movements. Especially in the process of physical confrontation, the importance of core strength training is self-evident, so that all links of the athlete's body can form a powerful whole, so as to ensure the coordination and flexibility between the upper and lower limbs, and improve the athlete's ability to use skills and tactics. Chao et al. believe that athletes need the participation of core areas in the process of making various difficult technical actions in training and competition. The core area plays an important role in the stability, coordination, and continuity of athletes in the process of completing various technical movements. They also proposed that the core strength area mainly refers to the lumbar and abdominal muscles, back muscles, hip muscles, and deeper muscle groups [8].

The article "Study on Strength and Quality Training of Youth Basketball Players" was retracted in 2023. Reasons: signs of a paper mill; suspected computer-generated content; unreliable results or conclusions; lack of ethics approval or compliance.

## 3. Athlete Training Monitoring System

### 3.1. Pneumatic Strength Training System

This paper studies a set of training equipment driven by air pressure as a load-bearing load [9]. This series of training equipment includes many horizontal equipment. Although each equipment has slightly different appearance and structure for different limb parts, the load source is all driven by air pressure, which is the same as training resistance. The training system studied in this topic includes two parts: the first level system is the service host for information storage and instruction distribution, and the second level system is the equipment directly involved in training, and its structure is shown in Figure 1.

As a service host, the primary system is carried on the PC side and is operated by the training center specialist to record and store data and issue training tasks. In terms of information exchange between the upper and lower systems, RFID wireless technology is integrated into each training mode with ID card as the medium, integrating the service system of the service host and the training needs of the training customers, so as to realize the real-time feedback analysis of training information.

### 3.2. Pneumatic Load Transfer Scheme

The scheme design of converting air pressure into load-bearing load mainly includes two aspects: on the one hand, the layout and structure of air pressure, on the other hand, the design logic of controlling air pressure, and at the same time, the mechanical structure of training equipment should be considered comprehensively in many aspects. As for the design of air circuit structure of air pressure perfusion, this research has high requirements for supplementing and unloading air pressure, which not only requires the control accuracy of proportional solenoid valve but also has corresponding requirements for the design structure of air circuit. After repeated tests, select the appropriate air pipe diameter and cylinder volume [10, 11]. The structure of pneumatic circuit is shown in Figure 2.

About the air pressure control, the embedded control system detects and adjusts the simulated load of the training equipment, that is, the air pressure value in the cylinder. During training, the sensor detects the air pressure value in the cylinder in real time and feeds it back to the master control to make corresponding adjustments. The design of pneumatic load feedback control of instruments and equipment is shown in Figure 3, forming a closed-loop control. The execution process of pneumatic load is as follows.

This research adopts the compound control of additional inverse model feedforward compensation and detecting current feedback PWM drive. In the PWM drive of proportional solenoid valve, in order to meet the control requirements at the same time, it is necessary to collect the current value on the coil at all times, and resistance is the simplest and most effective method, which is actually to adjust the deviation of the controlled quantity. It obtains the control deviation *e*(*t*) according to the present value *r*(*t*) and the test value *c*(*t*):

(1) $$\begin{array}{c} e\left(t\right)=r\left(t\right)-c\left(t\right). \end{array}$$

Then, taking *e*(*t*) as the input, the arithmetic unit performs PI and PD control. The output is as follows:

(2) $$\begin{array}{c} u\left(t\right)=Kp\left[e\left(t\right)+\frac{1}{Ti}\int_{0}^{t}e\left(t\right)dt+\frac{T_{d}de\left(t\right)}{dt}\right]+u_{0}\left(1\right). \end{array}$$

After conversion,

(3) $$\begin{array}{c} u\left(t\right)=Kpe\left(t\right)+K_{i}\int_{0}^{t}e\left(\tau \right)d\tau +K_{d}\frac{d}{dt}e\left(t\right)+u_{0}\left(1\right), \end{array}$$

where at time *t*, *u*(*t*) is the actual quantity, *e*(*t*) is the deviation, and *u*_0_ is the given value. Since STM32 is a digital component and belongs to discrete control, it should be discretized and converted into discrete state space expression:

(4) $$\begin{array}{c} u\left(KT\right)=K_{p}e\left(KT\right)+K_{i}\overset{k}{\underset{j=0}{\sum }}e\left(jT\right)+K_{d}\left[e\left(KT\right)-e\left(T\left(k-1\right)\right)\right]. \end{array}$$

In the above formula, *KT* is the number of time of the collected object, where *u*(*KT*) is the output value of the time [12],

*K*_*i*_ is the integral coefficient:

(5) $$\begin{array}{c} K_{i}=\frac{K_{p}T}{T_{i}}. \end{array}$$

*T*_*i*_ is the integral time constant.

The article "Study on Strength and Quality Training of Youth Basketball Players" was retracted in 2023. Reasons: signs of a paper mill; suspected computer-generated content; unreliable results or conclusions; lack of ethics approval or compliance.

*K*_*d*_ is the differential coefficient:

(6) $$\begin{array}{c} K_{d}=\frac{K_{p}T_{d}}{T}. \end{array}$$

*T*_*d*_ is the differential time constant.

In this pneumatic control system, the sampling frequency is jointly determined according to the air path aperture and the response speed of the proportional valve, as well as the air pressure feedback value in the cylinder, and then according to the deviation generated in the upper limb training process, the control quantity is calculated by proportion, integration, and differentiation for control. As for parameter setting, the critical proportional method is better than the failure curve method according to the control demand. The air pressure control of the trainer is adjusted at any time according to the specific requirements of the training equipment in the use process. The general operation flow chart of the training equipment is shown in Figure 4, and the specific steps are as follows [13, 14].

The training system has two methods to increase or decrease the air pressure load of the equipment:

- There is a mechanical addition button on the equipment shell to increase or decrease the load manually, and the size of the increase or decrease load is determined by the individual's will
- There is a control system that automatically replenishes or releases the load according to the feedback of the trainers, or when the system self-checks the equipment, it replenishes the load to reach the initialization value

The article "Study on Strength and Quality Training of Youth Basketball Players" was retracted in 2023. Reasons: signs of a paper mill; suspected computer-generated content; unreliable results or conclusions; lack of ethics approval or compliance.

### 3.3. Pneumatic Load Calibration

Due to the difference in the manufacturing process of the sensor, the air pressure value may correspond to different voltage values, and the detection voltage value provided to the main control will also be different. In order to ensure that the measured air pressure value and the detected and collected voltage value correspond correctly, the air pressure transmitter should be calibrated before use to determine the compensation, which is the significance of calibrating the initial value of the air pressure sensor. First, set the starting point and any point to determine the corresponding relationship between voltage and pressure. We select the initial value and the intermediate value (roughly determined) as 0 MPa and 0.3 MPa as the calibration standards, and set 0 MPa as the free state, that is, the atmospheric pressure. The output voltage of the sensor at 0 MPa is *a*, and the output voltage of the sensor at 0.3 MPa is *B* [15, 16]. The linear relationship between the collected voltage value and the detected pressure is as follows:

(7) $$\begin{array}{c} \text{Gas}P=\text{Gas}V*\frac{0.3\text{ MPa}}{B-A}. \end{array}$$

We set it as gross weight (*w*), which is the starting amount. According to physical mechanics, the load corresponding to air pressure is calculated as follows. *P* is the pressure in the cylinder, and *S* is the cross-section of the movable piston, where *K* is the weight proportion coefficient of the load. For this external instrument, that is, the ratio of the force on the cylinder piston to the force on the grip is pulled by the training customer. The purpose of adding the proportion coefficient is to eliminate the adverse effects such as friction. The weight of the load displayed on the LCD screen of the instrument is

(8) $$\begin{array}{c} W=P*S*K+w. \end{array}$$

Since the pneumatic simulator is used to load the machine, the above calculated tension value is the theoretical tension value FS. Then, we actually test the tension value of the bracelet grip as *F*_*C*_, and the relationship is shown in Figure 5 through actual repeated tests.

According to the experimental data, the measured arm tension *F*_*C*_ of the grip has the following relationship with the actual pressure Gas*P* in the cylinder, where *k* is the linear coefficient:

(9) $$\begin{array}{c} F_{C}=\text{Gas}P*k+2.1. \end{array}$$

In this paper, the diameters of the two proportional valves provided by KOFLOC3050 and KOFLOC3040 are selected, and the proportional solenoid valve is fitted and tested on the flow hysteresis curve according to the above fitting scheme. Two types of proportional valves were tested under 0.1 MPa air pressure. The air source was air, the input voltage was 24 V; the operation structure of the controller and the error parameters were obtained in the actual debugging [17]. Considering that this subject adopts incremental PID control, the calculation formula is

(10) $$\begin{array}{c} u\left(k\right)=u\left(k-1\right)+\Delta u\left(k\right), \end{array}$$

(11) $$\begin{array}{c} \Delta u\left(k\right)=K_{p}\left[e\left(k\right)-e\left(k-1\right)\right]+K_{I}\left(e\right)+K_{D}\left[e\left(k\right)-2e\left(k-1\right)+e\left(k-2\right)\right]. \end{array}$$

The magnitude of *K*_*p*_ directly determines the amplitude oscillation, and the amplitude oscillation will increase with the increase of *K*_*p*_ amplitude, but the oscillation frequency is small, and the system needs more time to achieve stability; *K*_*I*_ determines the action response speed, and *K*_*D*_ is used to eliminate static errors. Variables in the formula are as follows:

*e*(*k*): the error between the air flow through the flow valve and the theoretical value

*e*(*k* − 1): the error value of the previous time

*e*(*K* − 2): the error value of the previous sampling time

When |*e*(*k*)| is higher than the amplitude of PWM wave, the error is too large. At this time, the control quantity is directly output at the maximum value to reduce the error to the allowable range as soon as possible, where

(12) $$\begin{array}{c} \Delta u\left(k\right)=\Delta u_{\max}, \end{array}$$

(13) $$\begin{array}{c} \text{or }\Delta u\left(k\right)=-\Delta u_{\max}. \end{array}$$

At this time, the system is equivalent to implementing open-loop control. When *e*(*k*) · Δ*e*(*k*) ≥ 0, it means that it is a positive error at the moment, and the size of the error cannot be determined. The controller implements control, taking the absolute value of the reduced error as the control direction, and the controller output is as follows:

(14) $$\begin{array}{c} \Delta u\left(k\right)=K_{I}\left\{\begin{array}{c} K_{p}\left[e\left(k\right)-e\left(k-1\right)\right]+K_{I}e\left(k\right)\\ +K_{D}\left[e\left(k\right)-2e\left(k-1\right)+e\left(k-2\right)\right] \end{array}\right\}\;K_{I}>1. \end{array}$$

If |*e*(*k*)| is less than the set error limit, that is, the error is within the allowable range, there is no need for forced limit control, and general PID control can be implemented. When *e*(*k*) · Δ*e*(*k*) < 0 and *e*(*k*) · Δ*e*(*k* − 1) > 0, the control reduces the error to the equilibrium state and keeps the control unchanged, and the output is Δ*u*(*k*) = 0. When |*e*(*k*)| is less than a minimal positive number, the error is very small at this time. The controller adds integral control to reduce the steady-state error. The operation formula is proportional plus integral control:

(15) $$\begin{array}{c} \Delta u\left(k\right)=K_{p}\left[e\left(k\right)-e\left(k-1\right)\right]+K_{I}e\left(k\right). \end{array}$$

When *e*(*k*) = 0, it is proved that the system is basically error free at this moment and continues to maintain the current control relationship. After the fuzzy PID control processing of the variables by the master controller, the proportional valve drive circuit is driven by PWM wave, and the amplified PWM signal is supplied to the proportional valve to control the flow [18].

The article "Study on Strength and Quality Training of Youth Basketball Players" was retracted in 2023. Reasons: signs of a paper mill; suspected computer-generated content; unreliable results or conclusions; lack of ethics approval or compliance.

## 4. Comparative Study on Strength Quality Training of Juvenile Basketball Players

### 4.1. Research Design

#### 4.1.1. Research Object

In this article, a total of 20 members of the basketball special class of basketball school are selected as the experimental objects of this study. All of them are male teenagers aged 14-16 and have a certain foundation of professional basketball training. The basic information of each research object is shown in Table 1, and the basic physical information is shown in Figure 6.

#### 4.1.2. Experimental Method

The experiment period is from August 2020 to October 2020, and the training experiment lasts for 8 weeks. The duration of each experimental training should be controlled at about 35 minutes. In the training three times a week, the members of the experimental group wear pressure bandages for blood flow restriction training, while the members of the control group do not wear pressure bandages for traditional strength training (before the training officially begins, all experimental subjects need to carry out the pretest without blood flow restriction training device, and after all experiments, the posttest without blood flow restriction training device is required). Precautions and screening process before blood flow restriction training are shown in Figure 7.

Before the blood flow restriction training with a training load of 40% 1RM, the heart rate of the subjects was relatively flat, and there was no change in the heart rate after pressurization. After the blood flow restriction training for about 30 minutes, the immediate heart rate among the subjects did not fluctuate and deviate much, and the rate of heart rate recovery was basically the same as that of conventional resistance strength training [19].

### 4.2. Research Results and Analysis

#### 4.2.1. Comparison and Analysis of the Test Results of the Special Strength Quality of the Subjects before the Experiment

Before the formal experiment, the original data of 20 people in the four experimental groups were statistically analyzed by using the four strength quality indicators in the youth basketball special strength quality for this experiment. The mathematical statistics method is used to carry out the *t*-test of independent samples, and the one-way variance homogeneity test and ANVOA difference analysis are carried out uniformly, so as to ensure the scientificity and rationality of the selection of experimental objects and help to ensure the official start of the experiment and the smooth progress of the whole experimental cycle.

The article "Study on Strength and Quality Training of Youth Basketball Players" was retracted in 2023. Reasons: signs of a paper mill; suspected computer-generated content; unreliable results or conclusions; lack of ethics approval or compliance.

Before the official start of this experiment, four groups of experimental objects were tested to obtain the results, and the original data were passed through the one-way variance homogeneity test in SPSS mathematical statistics and ANVOA variance analysis to draw the conclusion, as shown in Table 2. Before the experiment was officially started, there was no significant difference between the three experimental groups and the control group in the 3RM test item of free bench press (*f* = 0.206, *p* = 0.891, *p* > 0.05). In the barbell free squat 3RM project (*f* = 0.118, *p* = 0.948, *p* > 0.05), there is no significant difference. In the 3/4 sprint events (*f* = 0.717, *p* = 0.556, *p* > 0.05), there is no significant difference. In 17(m) × 15(m) endurance turnaround runs, *f* = 0.088, *p* = 2.606, *p* > 0.05. In the test item of one-step vertical take-off and height touch on both feet, *f* = 1.821, *p* = 0.184. Among the above five items related to basketball special strength quality, the *p* value is greater than 0.05. There is no significant difference in special strength quality between the three experimental groups and the control group, and everyone's level is relatively similar.

From the data in Table 3, it can be concluded that the *T* value of the first group and the second group in the bench press 3RM test project is 0.188, the *p* value is 0.855 (*p* = 0.855), and *p* is greater than 0.05. There was no significant difference in the strength quality of bench press between the first group and the second group. The value of the independent sample *t*-test of the subjects of the first and third groups in the bench press 3RM project is *t* = −0.271 and *p* = 0.794, where *p* > 0.05, indicating that there is no significant difference between the two groups. The comparative analysis between the experimental group 1 and the traditional control group (*t* = 0.461, *p* = 0.657, *p* > 0.05) shows that there is no significant difference between the two groups before the official start of the experiment. After comparing the experimental group 2 with the experimental group 3, the conclusion is drawn as follows: *t* = −0.487, *p* = 0.639, and *p* > 0.05. There is no significant difference in the test results between the two groups. The comparison between the experimental group 2 and the traditional control group can be drawn as follows: *t* = 0.318, *p* = 0.759, and *p* > 0.05; there is no significant difference between the experimental group 2 and the control group. Finally, the comparison between the experimental group 3 and the control group shows that *t* = 0.318, *p* = 0.759, and *p* > 0.05. To sum up, experimental group 1, experimental group 2, experimental group 3, and the traditional control group have independent sample *t*-test, and the *p* value is greater than 0.05, which has no significant difference. The three groups of the experiment cross compare with each other, and the *p* value is also greater than 0.05. It is proved that there is no significant difference among 20 subjects in total between all groups in the 3RM maximum strength test of bench press before the start of the experiment, which meets the starting requirements of this experiment.

The article "Study on Strength and Quality Training of Youth Basketball Players" was retracted in 2023. Reasons: signs of a paper mill; suspected computer-generated content; unreliable results or conclusions; lack of ethics approval or compliance.

From the data in Table 4, it can be concluded that the *t* value of experimental group 1 and experimental group 2 in the squat 3RM test project is 0.352, *p* value is 0.734 (*p* = 0.734), and *p* is greater than 0.05. There is no significant difference in the strength quality of bench press between experimental group 1 and experimental group 2, while the value of independent sample *t*-test between experimental group 1 and experimental group 3 in the squat 3RM project is *t* = −0.04 and *p* = 0.969, where *p* > 0.05. It shows that there is no significant difference between the two groups. The comparison and analysis between the experimental group and the traditional control group (*t* = 0.436, *p* = 0.674, *p* > 0.05) show that there is no significant difference between the two groups before the official start of the experiment. After comparing the experimental group 2 with the experimental group 3, it is concluded that *t* = −0.399, *p* = 0.7, and *p* > 0.05; there is no significant difference in the test results between the two groups. Comparing the experimental group 2 with the traditional control group, it can be concluded that *t* = 0.67, *p* = 0.948, and *p* > 0.05; there is no significant difference between the experimental group 2 and the control group. Finally, the experimental group 3 is compared with the control group, and it is concluded that *t* = 0.488, *p* = 0.639, and *p* > 0.05. To sum up, experimental group 1, experimental group 2, experimental group 3, and the traditional control group have independent sample *t*-test, and the *p* value is greater than 0.05, which has no significant difference. The three groups of the experiment cross compare with each other, and the *p* value is also greater than 0.05. It is proved that there is no significant difference among 20 subjects in total between all groups in the squat 3RM maximum strength test before the start of the experiment, which meets the starting requirements of this experiment [20].

The article "Study on Strength and Quality Training of Youth Basketball Players" was retracted in 2023. Reasons: signs of a paper mill; suspected computer-generated content; unreliable results or conclusions; lack of ethics approval or compliance.

After the 8-week training experiment, the paired sample *t*-test in the SPSS statistical software was used to calculate and compare the test results of the four test indicators selected from the basketball special strength quality of boys in the traditional control group before and after the experiment, so as to verify the changes and effects of traditional special resistance strength training compared with blood flow restriction training on the basketball special strength quality of young basketball players. The results are shown in Table 5.

Moreover, on the premise of not carrying out the training of wearing compression devices, the effect of the traditional control group has a large gap compared with the three experimental groups in terms of the pre- and postcomparison results of bench press and squat events. The degree of improvement of the control group before and after the training was about 4.8 kg, which was very balanced and regular. Perhaps because it did not carry out the same heavy and high-intensity load training as the traditional resistance strength training, it led to the improvement, but compared with the three experimental groups of blood flow restriction training, it did not have satisfactory effect.

#### 4.2.2. Comparative Analysis of the Test Results of the Maximum Strength Quality in Basketball Special Strength Quality after the Experiment

After the experiment of blood flow restriction basketball special strength training three times a week for eight weeks, a postexperiment test was carried out for a total of 20 subjects in four groups in the experiment after the experiment was completed and the four test indicators of teenagers' basketball special strength in the postexperiment test. In order to further explore the relationship between these indicators among the four groups participating in this experimental training, the SPSS statistical software will be used to conduct one-way ANOVA and independent sample *t*-test on all the original data of the postexperimental test, analyze the relationship between the test data of different strength qualities in different groups, and analyze and discuss the reasons for the changes of these data. The specific results are shown in Table 6.

The article "Study on Strength and Quality Training of Youth Basketball Players" was retracted in 2023. Reasons: signs of a paper mill; suspected computer-generated content; unreliable results or conclusions; lack of ethics approval or compliance.

As shown in Table 7, after 8 weeks of blood flow restriction basketball special strength training, the average value of the bench press 3RM test of the experimental group 1 was 65.2 kg, that of the experimental group 2 was 65.7 kg, that of the experimental group 3 was 72.2 kg, and that of the traditional control group was 55.4 kg. Among them, experimental group 2 has an advantage of 0.5 kg compared with experimental group 1, experimental group 3 has an advantage of 7 kg compared with experimental group 1, and experimental group 2 has a disadvantage of 6.5 kg compared with experimental group 3, while the traditional control group has a disadvantage of 9.8 kg compared with experimental group 1, 10.3 kg compared with experimental group 2, and 16.8 kg compared with experimental group 3.

In the one-way variance test results of the 3RM item of bench press in the relevant special strength quality after the experiment is completed, *f* = 6.403. Next, we can see that the later *p* value is 0.005, *p* < 0.01, indicating that there is an extremely significant difference between the four groups of bench press after the experiment has trained eight groups. Next, it can be seen from Table 7 that the *p* value of the experimental group 1 and experimental group 2 is 0.855, and the mean difference is 0.5 kg, indicating that the training effect of bench press quality in low-intensity compression group and medium-intensity compression group is roughly the same after eight weeks of training, and there is no significant difference. The *p* value of the first group and the third group is 0.145, and the mean difference is 7 kg. The mean difference between the second group and the third group is 6.5 kg. Look back at the mean difference between the first group and the second group. The test results of the three groups are compared with each other, which shows that although the difference between the low-intensity pressure group and the high-intensity pressure group is still not significant, there is a relatively obvious gap compared with the medium pressure group. It also preliminarily shows that within the safe and reasonable range of values, with the continuous increase of the pressure load, the performance of the recumbent push of the athletes who carry out blood flow restriction basketball special strength training will also be improved more significantly.

By analyzing the bench press performance of the three experimental groups and the traditional control group, the average difference between the experimental group 1 and the traditional control group is 9.8 kg, the difference between the experimental group 2 and the traditional control group is 10.3 kg, and the difference between the experimental group 3 and the traditional control group has reached an amazing 16.8 kg. However, the *p* values obtained by the experimental group 2 and the experimental group 3 and the control group are all less than 0.05, and the *p* values obtained by the experimental group 3 have been less than 0.01, which is still significantly improved compared with the traditional control group, and the *p* values also decreased significantly compared with those before the experiment. This shows that under the same training load, the same interval time between groups and the same training plan, compared with the traditional resistance strength training, the blood flow restriction training has a very obvious improvement and progress in the strength quality of bench press 3RM of juvenile basketball players in basketball school. And under different pressure load conditions, the same training results will be different. The performance of bench press will increase with the increasing pressure value, and there is a positive correlation between the two.

The article "Study on Strength and Quality Training of Youth Basketball Players" was retracted in 2023. Reasons: signs of a paper mill; suspected computer-generated content; unreliable results or conclusions; lack of ethics approval or compliance.

## 5. Conclusion

This paper combines the blood flow restriction training method with basketball special strength training, in order to explore the advantages of this training method for young basketball players' special strength quality, compared with the traditional resistance strength training, and the changes in body shape and function. This paper attempts to provide some references and suggestions for the training plan of the combination of the two and the optimization of the pressure value within the safe range of pressure application. Through the research, it is found that (1) blood flow restriction training can effectively improve the special strength quality of juvenile basketball players in basketball school, and it is the most significant to improve the maximum strength quality and strength endurance quality, which is significantly better than the control group. Although the speed strength and explosive force quality have been improved, the effect is not obvious, and the explosive force quality effect of the high pressure load group is less than that of the control group; (2) blood flow restriction training can effectively improve the cardiopulmonary function of juvenile basketball players. The heart rate decreased in quiet state, and the rate of heart rate returning to calm increased after exercise, indicating that blood flow restriction training enhanced the pumping function of the heart and indirectly improved the adaptability of muscles to high load intensity training; (3) through the test, it is found that the experimental group has a significant effect on the improvement of maximum strength no matter whether it compares itself before and after or with the control group. For strength endurance, explosive force, and speed force, the greater the pressure load, the better the effect. It shows that within the scientific and safe pressure range, the greater the pressure on the body, the better the training effect. Appropriate pressure value and interval time, as well as more targeted training programs, can achieve twice the result with half the effort compared with traditional resistance strength training.

The article "Study on Strength and Quality Training of Youth Basketball Players" was retracted in 2023. Reasons: signs of a paper mill; suspected computer-generated content; unreliable results or conclusions; lack of ethics approval or compliance.

Of course, it is necessary to make necessary preparations before trying blood flow restriction training. Before training, fully prepare for the preparatory activities and special warm-up exercises, and then carry out the adaptive activities of blood flow restriction training, and timely report to the coach whether the blood flow restriction training device is suitable and stable, as well as whether the physical condition of the experimental object is uncomfortable in the process of gradually increasing pressure. It is suggested that the team members who first try blood flow restriction training should be equipped with team doctors for real-time monitoring and risk and safety assessment, so as to ensure the health of the team members and prevent accidents. After blood flow restriction training, the pressure band must be removed as soon as possible with the guidance and help of the coach and team doctor. It is recommended to use various physical means to relax and stretch after strength training after the blood pressure and heart rate return to the normal range. To prevent excessive lactic acid accumulation and fascia adhesion, which will affect the training effect, it is suggested to carry out comparative training according to the flow chart of blood flow restriction training safety strategy, so as to ensure the scientific and safe training content.

## Figures and Tables

**Figure 1:** System operation structure.

**Figure 2:** Pneumatic circuit structure.

**Figure 3:** Pneumatic load control flow chart.

**Figure 4:** Operation process of solenoid valve.

**Figure 5:** Comparison between theoretical tension and measured tension.

**Figure 6:** Basic physical conditions of objects in basketball special class of basketball school.

**Figure 7:** Flow chart of selecting pressure training strategy.

**Table 1:** Basic information of experimental objects in basketball special class of basketball school.

Age	Height (cm)	Weight (kg)	BMI
16	180	75	23.1
16	190	85	23.5
14	179	70	21.8
16	179	72	22.4
15	182	65	19.6
16	174	71	20.9
14	180	76	23.4
14	177	70	22.3
16	176	72	23.2
16	180	68	20.9
16	178	72	22.7
14	186	70	20.2
16	183	77	22.9
16	174	81	23.9
16	185	74	21.6
16	186	83	23.9
16	195	86	22.6
15	182	71	21.4
16	192	82	22.2
14	187	73	20.8

The article "Study on Strength and Quality Training of Youth Basketball Players" was retracted in 2023. Reasons: signs of a paper mill; suspected computer-generated content; unreliable results or conclusions; lack of ethics approval or compliance.

**Table 2:** One-way ANOVA of special strength indicators of subjects before the experiment.

*N* = 5	Bench press 3RM (kg)	Squat 3RM (kg)	3/4 full court run (s)	17 × 15 running (s)	Jump and touch high (cm)
Experiment group 1	53.2 ± 9.31	69.6 ± 8.26	4.08 ± 0.34	74.01 ± 4.89	315.60 ± 7.23
Experiment group 2	52.2 ± 7.36	67.6 ± 9.65	3.82 ± 0.48	66.89 ± 4.01	310.20 ± 7.46
Experimental group 3	54.8 ± 9.39	69.8 ± 7.66	3.91 ± 0.31	72.29 ± 4.91	309.00 ± 9.30
Control group	50.6 ± 8.50	67.2 ± 9.12	3.78 ± 0.26	70.71 ± 2.58	318.00 ± 2.91
*p*	0.891	0.948	0.556	2.606	1.821
*f*	0.206	0.118	0.717	0.088	0.184

**Table 3:** Multiple interactive comparative analysis of bench press items in the special strength of the subjects before the experiment.

Comparison group A	Comparison group B	Bench press 3RM mean ± standard deviation (kg)		*t* value	*p* value
Experiment group 1	Experiment group 2	53.2 ± 9.31	52.2 ± 7.36	0.188	0.855
Experiment group 1	Experimental group 3	53.2 ± 9.31	54.8 ± 9.39	-0.271	0.794
Experiment group 1	Control group	53.2 ± 9.31	50.6 ± 8.50	0.461	0.657
Experiment group 2	Experimental group 3	52.2 ± 7.36	54.8 ± 9.39	-0.487	0.639
Experiment group 2	Control group	52.2 ± 7.36	50.6 ± 8.50	0.318	0.759
Experimental group 3	Control group	54.8 ± 9.39	50.6 ± 8.50	0.741	0.480

**Table 4:** Multiple interactive comparative analysis of squat items in the special strength of the subjects before the experiment.

Comparison group A	Comparison group B	Squat 3RM mean ± standard deviation (kg)		*t* value	*p* value
Experiment group 1	Experiment group 2	69.6 ± 8.26	67.6 ± 9.65	0.352	0.734
Experiment group 1	Experimental group 3	69.6 ± 8.26	69.8 ± 7.66	-0.040	0.969
Experiment group 1	Control group	69.6 ± 8.26	67.2 ± 9.12	0.436	0.674
Experiment group 2	Experimental group 3	67.6 ± 9.65	69.8 ± 7.66	-0.399	0.700
Experiment group 2	Control group	67.6 ± 9.65	67.2 ± 9.12	0.670	0.948
Experimental group 3	Control group	69.8 ± 7.66	67.2 ± 9.12	0.488	0.639

**Table 5:** Comparative analysis of special strength indicators of traditional control group.

*N* = 5	Bench press 3RM (kg)	Squat 3RM (kg)	3/4 full court run (s)	17 × 15 run (s)	Vertical jump height (CM)
Before experiment	50.6 ± 8.50	69.6 ± 8.26	3.782 ± 0.257	70.71 ± 2.58	318.0 ± 2.91
Eight weeks of experiment	55.4 ± 7.34	74.7 ± 6.96	3.678 ± 0.256	69.35 ± 2.04	319.6 ± 2.30
*p*	0.082	0.058	0.007	0.630	0.016
*f*	-2.311	-2.627	5.039	2.561	-4.000

**Table 6:** One-way ANOVA of the 3RM test results of bench press in basketball special strength quality after the experiment.

Control group (*N* = 5)	Mean ± standard deviation (kg)	Homogeneity test	*f* value	*p* value
Experiment group 1	65.2 ± 5.76			
Experiment group 2	65.7 ± 1.39	0.600	6.403	0.005
Experiment group 3	65.7 ± 1.39			
Traditional control group	55.4 ± 7.34			

The article "Study on Strength and Quality Training of Youth Basketball Players" was retracted in 2023. Reasons: signs of a paper mill; suspected computer-generated content; unreliable results or conclusions; lack of ethics approval or compliance.

**Table 7:** Independent sample *t*-test analysis table of 3RM test results of bench press in basketball special strength quality after the experiment.

Group A	Group B	Mean difference	*t* value	*p* value
Experiment group 1	Experiment group 2	-0.5	-0.189	0.855
Experiment group 1	Experimental group 3	-7.0	-1.614	0.145
Experiment group 1	Traditional control group	9.8	2.348	0.470
Experiment group 2	Experiment group 3	-6.5	-1.834	0.104
Experiment group 2	Traditional control group	10.3	3.081	0.015
Experiment group 3	Traditional control group	16.8	3.507	0.008

## Data Availability

The labeled data set used to support the findings of this study is available from the corresponding author upon request.
